The article "Characterization and Dynamic Behavior of Wild Yeast during Spontaneous Wine Fermentation in Steel Tanks and Amphorae" was published in 2013. Journal: Biomed Res Int.

# Characterization and Dynamic Behavior of Wild Yeast during Spontaneous Wine Fermentation in Steel Tanks and Amphorae

**DOI:** 10.1155/2013/540465

**Published:** 2013-05-02

**Authors:** Cecilia Díaz, Ana María Molina, Jörg Nähring, Rainer Fischer

**Affiliations:** ^1^Molecular Biology Division, Fraunhofer Institute for Molecular Biology and Applied Ecology, 57392 Schmallenberg, Germany; ^2^Facultad de Ingeniería y Tecnología, Universidad San Sebastián, 4030000 Concepcion, Chile

## Abstract

We studied the dynamic behavior of wild yeasts during spontaneous wine fermentation at a winery in the Valais region of Switzerland. Wild yeasts in the winery environment were characterized using a PCR-RFLP method. Up to 11 different yeast species were isolated from the vineyard air, whereas only seven were recovered from the grapes surface. We initially investigated a cultureindependent method in pilot-scale steel fermentation tanks and found a greater diversity of yeasts in the musts from two red grape varieties compared to three white grape varieties. We found that the yeasts *Metschnikowia pulcherrima*, *Rhodotorula mucilaginosa*, *Pichia kluyveri*, *P. membranifaciens* and *Saccharomyces cerevisiae* remained active at the end of the fermentation. We also studied the dynamic behavior of yeasts in Qvevris for the first time using a novel, highlysensitive quantitative real-time PCR method. We found that non-*Saccharomyces* yeasts were present during the entire fermentation process, with *R. mucilaginosa* and *P. anomala* the most prominent species. We studied the relationship between the predominance of different species and the output of the fermentation process. We identified so-called spoilage yeasts in all the fermentations, but high levels of acetic acid accumulated only in those fermentations with an extended lag phase.

## 1. Introduction

Low-intervention winemaking methods based on spontaneous fermentation are becoming more popular among wine producers and consumers [1, 2]. Some wine producers and viticulturists have readopted traditional winemaking methods to generate unique attributes that differentiate their products, improve wine quality, and increase the variety of complex flavors that characterize regional vineyards.

Spontaneous fermentation is a complex process influenced by many factors, including the endogenous microbial flora, the grape variety, climatic conditions, and the winemaking process [3–7]. The outcome of the fermentation process can therefore be difficult to predict and can differ from year to year. The natural yeast flora, found on grapes and in wineries, play a significant role during fermentation and are particularly important during spontaneous fermentation because no additional wine yeasts are introduced into the process.

Wine flavor is influenced by the large number of yeast species present during spontaneous fermentation [3, 8–11], including those from the genera *Hanseniaspora*, *Metschnikowia* and *Candida*, and more occasionally *Torulaspora* and *Pichia*. Most of these non-*Saccharomyces* yeasts grow during the early fermentation stages, whereas the process is eventually completed by *Saccharomyces cerevisiae* because it can tolerate higher levels of alcohol and lower levels of oxygen [9–15].

Previous studies have shown that non-*Saccharomyces* yeasts can be detected throughout the fermentation process [15]. They influence the course of fermentation and the characteristics of the resulting wine by producing extracellular enzymes and metabolites of oenological significance that modify the sensory and organoleptic properties of wine, introducing a broader spectrum of aromas and flavors [16–18].

Microbiology techniques are often used to isolate and identify wild yeasts, but this requires different types of media and different culture protocols that influence species which are recovered. The metabolic status of the cells also results in the presence of viable but nonculturable (VBNC) microbes whose influence on fermentation can be underestimated because the population dynamics cannot be evaluated accurately. Quantitative real-time PCR (qPCR) is a faster and more reliable alternative to identify and quantify yeasts during fermentation [19] and is particularly advantageous for VBNC yeasts because of its sensitivity [20]. Although the technique cannot distinguish living cells from intact dead cells, it remains the most widely used method for the evaluation of wild yeast dynamics during fermentation because VBNC cells continue to influence wine flavor and palatability regardless of their actual status [21]. 

We compared microbiology methods (viable counts) and novel molecular biology techniques: polymerase chain reaction/restriction fragment length polymorphism (PCR-RFLP) and qPCR for the identification of yeast species, and we characterized their dynamic behavior during spontaneous wine fermentation in the Valais region of Switzerland in the 2008–2011 harvests. We used these new methods to identify the predominant species present during spontaneous fermentation, establishing a standard for the semiquantitative detection of yeasts with antibodies in a biochip format. Such a device would allow winemakers to make early decisions about the suitability of grapes and the likely success of spontaneous fermentation. Also for the first time, we studied the dynamic behavior of wild yeasts during spontaneous fermentation in Qvevris (amphora-like clay vessels), the use of which is an emerging trend among European winemakers.

## 2. Materials and Methods

### 2.1. Samples

Grapes and must samples were collected from the vineyards of the winery Albert Mathier et Fils S.A., in Salgesch, Valais, Switzerland, during the 2008–2011 harvest seasons. The grape varieties we studied are listed in Table 1. Samples were collected *in situ* and frozen at −20°C during transport prior to analysis. 

### 2.2. Isolation of Yeasts from the Winery Environment and Fermentation Samples

During 2008 and 2009, we screened yeasts present in the winery environment (i.e., the vineyard, winery facilities and cellar) and in the fermenting wine musts. In the vineyard, grape berries were placed in direct contact with plates containing Rose Bengal Chloramphenicol Agar (RBCA), a selective medium for yeasts and molds (15 g L^−1^ agar, 10 g L^−1^ glucose, 5 g L^−1^ papain-digested soybean meal, 1 g L^−1^ KH_2_PO_4_, 0.5 g L^−1^ MgSO_4_  × 7H_2_O, 0.05 g L^−1^ Rose Bengal, and 10 g L^−1^ chloramphenicol). We pumped 1000 L of vineyard air surrounding the grapes through a Millipore M Air Tester T (Millipore, USA) and plated the collected residue on RBCA as above. We also sampled environmental yeast flora from the winery facilities. Contact samples were taken from the inner surface of clean fermentation tanks before filling them with grape juice, and 1000 L of air inside the cellar was also filtered and the collected residues were plated as above. All the environmental samples were collected in triplicate.

Five different grape varieties from the 2008-2009 harvests (Table 1) were processed by spontaneous fermentation to determine the predominant yeast species at the different fermentation stages. Prefermentation steps such as harvesting and pressing were carried out according to routine winery procedures. Pressed berries were fermented with the skin to make red wine, or were clarified before fermentation to produce white wine. Duplicate fermentations were carried out in the winery cellar using new 110-L stainless steel tanks, without starting yeast cultures. Liquid samples (50 mL, in duplicate) from the fermenting musts were collected daily, frozen immediately at −20°C, and stored in the dark prior to analysis. Immediately after defrosting, liquid samples were centrifuged at 4000 rpm for 5 min. The supernatant was tested for chemical parameters, and the pellet was resuspended in 100 *μ*L distilled water, plated on RBCA medium and incubated at 30°C for 3–7 days, and then stored at 4°C prior to analysis.

### 2.3. Fermentation Parameters

The fermentations were monitored by measuring glucose/fructose consumption and ethanol formation during fermentation, and the acetic acid content at the end of fermentation. The parameters were determined by spectrophotometry at 20 ± 1°C using the D-Glucose/D-Fructose, Ethanol, and Acetic Acid enzymatic kits provided by R-Biopharm (Germany), according to the manufacturer's instructions. Standards and controls were provided in the kits. All measurements (duplicate fermentations) were taken in triplicate. 

### 2.4. Identification of the Predominant Yeast Species

A terminal restriction fragment length polymorphism (T-RFLP) method was developed and optimized for yeast identification, based on restriction patterns generated from the genomic region spanning the internal transcribed spacers (ITS1 and ITS2) and the 5.8S rRNA gene. These regions show low intraspecific polymorphism and high interspecific variability and have previously been shown to distinguish 26 yeast species found on grapes, in cellars and/or in wine musts [22, 23].

Total DNA from the isolated colonies was extracted using the First-Beer Magnetic DNA kit (GEN-IAL GmbH, Troisdorf, Germany) and amplified using primers ITS-5 (5′-GGA AGT AAA AGT CGT AAC AAG G-3′) and ITS-4 (5′-TCC TCC GCT TAT TGA TAT GC-3′) followed by a second round of amplification with the nested primers ITS-1 (5′-TCC GTA GGT GAA CCT GCG G-3′) and ITS-2 (5′-GCT GCG TTC TTC ATC GAT GC-3′) [24]. The first reaction mixture comprised 200 *μ*M of each dNTP, 10x PCR buffer, 0.5 *μ*M of each primer, 1 *μ*L of extracted yeast DNA and 1.25 U Hot Start Polymerase (5 Prime, Hamburg, Germany) in a total volume of 25 *μ*L. The samples were amplified in a thermocycler (VRW, Pennsylvania, USA) by denaturing at 95°C for 3 min followed by 15 cycles of denaturing at 95°C for 30 s, annealing at 57°C for 30 s and extension at 72°C for 1 min, and a final extension step at 72°C for 5 min. The nested amplification mixture comprised 200 *μ*M of each dNTP, 10x PCR buffer, 0.5 *μ*M of each primer (labeled if necessary for product size determination, see below), 2.5 U Hot Start Polymerase (5 Prime, Hamburg, Germany), and 0.5 *μ*L template DNA (from the first-round PCR) in a total volume of 50 *μ*L. The mixture was denatured at 95°C for 3 min then amplified by 20 cycles of denaturing at 95°C for 30 s, annealing at 62°C for 30 s and extension at 72°C for 1 min, followed by a final extension at 72°C for 5 min. The products were digested with BstYI (New England BioLabs, Ipswich) at 60°C for 1 h. The length of the terminal fragment was determined using a 3130 Genetic Analyzer (Applied Biosystems, Darmstadt, Germany) prior to the purification of the samples using the Cycle Pure Kit (Omega Bio-tek, USA).

### 2.5. Primer Design and Real-Time PCR

Primers specific for the 10 predominant yeasts found in the winery and in fermentation samples during the 2008-2009 harvest season were designed to anneal within the 26S rDNA region and amplify products 150–200 bp in length (Table 2). Each primer pair was designed by processing available sequences using CLC Combined Workbench 3 Software (CLC-Bio, Denmark), and the properties of each primer were verified using Primer Tool (Sigma-Aldrich, USA; http://www.sigmagenosys.com/calc/DNACalc.asp). The specificity of each primer pair was controlled by searching GenBank using BLAST (http://www.ncbi.nlm.nih.gov/BLAST/).

Real-time PCR was carried out using an ABI 7300 Real-Time PCR System (Applied Biosystems, Hitachi, Japan). Each reaction comprised 7.5 *μ*L Platinum SYBR Green qPCR SuperMix-UDG (Bio-Rad, Hercules, CA, USA), 200 nM of each primer (Metabion, Germany), and 0.3 *μ*L template DNA extracted from must, in a total volume of 15 *μ*L. The mixture was heated to 50°C for 2 min and then 95°C for 2 min, followed by 40 cycles of denaturation at 95°C for 15 s, and annealing/extension at 60–63°C (depending on the primers) for 45 s. The cycling temperature was then increased by 0.3°C every 10 s from 63 to 95°C to obtain the melting curve. The DNA concentration in the samples was limited to 50 ng per analysis, except for standard curves prepared from samples containing a known number of yeast cells. All yeast species were cultivated in Yeast Extract Peptone Dextrose (YPD) agar (10 g L^−1^ yeast extract, 20 g L^−1^ peptone, 20 g L^−1^ glucose, and 0.1 mg L^−1^ chloramphenicol) at 27°C for 24 h. The cells were counted using a Neubauer chamber. DNA was extracted using the First-Beer Magnetic DNA kit and serially diluted (1 : 10) from 10^7^-10^8^ down to 1 cell mL^−1^. Each point on the calibration curve was measured in duplicate. Conventional and real-time PCR was carried out using a range of yeast species to verify the specificity of each primer set. 

### 2.6. Wild Yeast Dynamics during Spontaneous Fermentation in Qvevris

Spontaneous fermentation in Qvevris was studied during the 2010 and 2011 harvest seasons. The white grape varieties Resi and Ermitage (Table 1) were harvested, crushed, and fermented in 1500-L Qvevris without clarification. We took 50-mL samples in triplicate at 2-3-day intervals throughout fermentation; that is, every time the Qvevris were opened to stir the must. The samples were frozen immediately at −20°C and stored in the dark prior to analysis. DNA was extracted from the must using a modified CTAB method [25] in which 10 mL samples were centrifuged for 1 min at 3000 rpm to sediment the skin and seeds before the standard protocol was applied. The extracted DNA was then tested by qPCR to identify the wild yeast species present during spontaneous fermentation as discussed above.

## 3. Results

### 3.1. Establishing a PCR-RFLP Method for Yeast Identification

Yeast genomic DNA was amplified using primers ITS4 and ITS5 (first round), and the products were amplified with the nested primers ITS1 and ITS2. The sizes of both the digested and undigested PCR products are unique to particular yeast genera and also allow the differentiation of certain species, resulting in the unambiguous identification of up to 28 species (Table 3). There were only three cases in which we were unable to distinguish two different species: (1) *Hanseniaspora guilliermondii* and *H. uvarum*; (2) *Saccharomyces bayanus* and *S. pastorianus*; (3) *Dekkera bruxellensis* and *Cryptococcus flavus*. The method was optimized using species obtained from the Deutsche Sammlung von Mikroorganismen und Zellkulturen GmbH (DSMZ), Braunschweig, Germany. Even so, wild yeast species in wineries are often local subspecies that are subject to different environmental selection conditions and their sequences and PCR product sizes can differ slightly from purchased strains. Therefore, and in order to validate the method, we selected 4 isolated yeasts and sequenced the first-round PCR products (NCBI accession numbers KC869927, KC869928, KC869929, and KC869930) to compare these empirical sequences to those in GenBank by using the empirical sequences as BLAST queries.

### 3.2. Natural Flora in Vineyard and Cellar Environments

Yeasts naturally present in the vineyard environment were isolated from the grape surface and from the air around the grapes using culture-dependent methods (see Section 2.2). During 2008 and 2009, up to 11 different yeast species could be isolated from the vineyard air although *Bulleromyces albus* and *Sporidiobolus pararoseus* were the only species recovered in both years (Table 4). We recovered seven yeast species from the grape surface, and species appear to be dependent on the variety and the year of harvest (Table 4). *Aurebasidium pullulans*, *Cryptococcus magnus*, *Rhodotorula mucilaginosa,* and *Zygosaccharomyces florentinus* were the only species isolated from both the air and the grape surface. Most of the yeasts isolated from the vineyard air were also present in the grape juice at the beginning of fermentation. In the cellar environment, yeasts were isolated from the surface of clean and empty barrels (i.e., before filling the fermentation tanks with the grape must) and from the air inside the cellar room. In 2008, four different species were isolated from the cellar air and three from the clean fermentation tank (Table 4), whereas in 2009 only one species (*R. mucilaginosa*) was isolated from the clean fermentation tank. All the species in the cellar environment were also found in the vineyard, and all species identified in the cellar environment were also later found in the fermenting must.

### 3.3. Yeast Flora in Steel-Tank Fermentations

Changes in the composition of the yeast population during spontaneous fermentation in steel tanks were measured using culture-dependent methods. We investigated the musts of five grape varieties during the 2008 and 2009 harvest seasons: the red varieties Pinot Noir and Cornalin, which contained 12 and 9 different yeast species, respectively, and the white varieties Gutedel, Chardonnay, and Petite Arvine, which contained 12, 12, and 7 yeast species, respectively (Table 5). 

Most of the yeast species we identified were present in more than one of the musts (Table 5). *M. pulcherrima*, *S. cerevisiae*, *S. bayanus,* and *T. delbrueckii* were found in all five musts at some point during fermentation. Six yeast species were only found in one type of must, and only at the beginning of fermentation. Four yeast species found in Gutedel musts did not grow in any of the other musts: *Bulleromyces albus*, *Candida zeylanoides*, *Cryptococcus flavus/Dekkera bruxellensis* (the latter could not be distinguished on the basis of their PCR-RFLP patterns), and *Filobasidium floriforme*. Similarly, *Pichia burtonii* and *P. holstii* only found in Cornalin musts (Table 5). There were no species associated exclusively with red or white grape varieties.

The composition of the yeast populations also changed significantly during fermentation. Initially, 7–12 different species were found in the musts (depending on the variety), but this declined to 1–5 species by the midfermentation, when nitrogen becomes limiting and the ethanol concentration begins to increase rapidly (Table 5). By the end of fermentation, only six different yeast species could be recovered from the musts. The ethanol-resistant strain *S. bayanus* made up a substantial proportion of the yeasts in all musts (Figure 1) and was the only strain detected in Gutedel musts during the mid- and late fermentation stages. In contrast, *S. cerevisiae* was found in the Chardonnay, Pinot Noir, and Petite Arvine musts at the end of fermentation, and *M. pulcherima* was present in the Chardonnay, Pinot Noir, and Cornalin musts at the end of fermentation. The other species retrieved at the end of the fermentation were *P. klyveri* (Chardonnay and Cornalin musts), *P. membranifaciens *(Chardonnay must), and *R. mucilaginosa* (Pinot Noir must) (Figure 1).

The progress of fermentation was monitored by measuring sugar consumption and ethanol production (Figure 2), as well as acetic acid production (Table 6). The red varieties Pinot Noir and Cornalin reached dryness (less than 4 g L^−1^ of total sugar) 6–11 days after pressing (Figure 2). The lag phase of the Pinot Noir fermentations in 2008 (i.e., the period before glucose consumption increases rapidly) was relatively long compared to the Cornalin fermentations in the same year (2-3 days) (Figure 2). In contrast, the white grape varieties failed to reach dryness in fermentations during 2008 and 2009, and the Petite Arvine and Chardonnay vessels contained high levels of residual sugar at the end of fermentation (Figure 2). In 2008, the fermentation of Gutedel grapes was delayed at the midexponential phase (days 6–13) whereas Petite Arvine was characterized by sluggish fermentation from the late exponential phase (day 11) onwards (Figure 2). 

### 3.4. Real-Time PCR

Thirteen pairs of specific primers were designed for the rapid identification and quantification of the yeast species we detected. The primers designed for *Z. florentinus*, *C. glabrata,* and *P. fermentans* showed evidence of nonspecific annealing and were therefore eliminated from the study. The sequences and annealing temperatures of the remaining primers are summarized in Table 2. The melt curve analysis for each PCR showed a single peak (data not shown). Standard curves were established for each pair of primers. The reaction efficiencies ranged between 72.54% (*P. anomala*) and 98.68% (*S. cerevisiae*) with high reproducibility. The lowest detection limit was 10^2^ cells L^−1^. 

### 3.5. Yeast Flora in Qvevri Fermentations

The dynamic behavior of the yeast populations in Qvevri spontaneous fermentations was monitored by qPCR during the 2010 and 2011 harvest seasons. There was a slight tendency towards higher yeast diversity in the Resi variety compared to Ermitage, with 10 and 8 different yeast species, respectively (Table 7). Most of the species were present in varieties, and *M. pulcherima, R. mucilaginosa, P. anomala, H. uvarum, S. cerevisiae,* and *T. delbrueckii* were also found at every fermentation stage (Figures 3 and 4). In contrast, *C. zemplinina* and *P. angusta* were found only in the Resi variety, and although *P. kluyveri* was found in both varieties, it was present only at certain fermentation stages during the 2010 harvest and was not detected in 2011 (Table 7). 

*R. mucilaginosa* was the dominant species in the 2011 Ermitage fermentations whereas *P. anomala* was the dominant species in the Resi fermentations in both harvest years. Up to eight yeast species were detected in the Ermitage fermentations during 2010 and 2011 (Table 7), and in both cases the dominant species in the must before fermentation were *R. mucilaginosa,* and *P. anomala* although they were more abundant in 2011 (Figure 3). The less-abundant species were *H. uvarum*, *S. cerevisiae*, *T. delbrueckii,* and *C. zemplinina*, although all of them were present throughout the fermentation. These species were 10 times more abundant in 2010 than in 2011, except *R. mucilaginosa*, which was more abundant in 2011. *S. cerevisiae* was the most abundant species at the beginning of the 2010 fermentations and it proliferated rapidly, reaching its maximum concentration (1 × 10^6^ cells mL^−1^) by day 6. In contrast, *R. mucilaginosa* was the most abundant species in the 2011 fermentations (1 × 10^6^ cells mL^−1^) and *S. cerevisiae* proliferated more slowly, reaching its maximum concentration after 14 days. In 2010, the yeast population declined slowly during fermentation whereas in 2011 the *P. anomala*, *S. cerevisiae,* and *R. mucilaginosa* populations remained high (Figure 3).

The Resi fermentations during 2010 and 2011 began rapidly (before 5 days in both cases) with *P. anomala* dominating throughout fermentation and *H. uvarum* and *T. delbrueckii *present at lower levels (Figure 4). The concentration of yeast, including *S. cerevisiae*, was slightly higher in 2010 than 2011 although the onset of fermentation in 2011 was more rapid, beginning after 1 day (Figure 4). In 2010, the highest concentration of *S. cerevisiae* (1 × 10^6^ cells mL^−1^) was achieved 2 days after fermentation began, whereas in 2011 the concentration increased rapidly during the first day and remained high until the end of the fermentation (1 × 10^6^ cells mL^−1^). 

The progress of the Ermitage and Resi fermentations was monitored and compared. The onset of the Ermitage fermentation took longer in 2010 but was nevertheless complete after 14 days in both 2010 and 2011 (Figure 5). The Ermitage fermentations did not reach dryness by day 14 in 2011, and the ethanol content was lower than in the 2010 fermentation, concomitant with the production of significant amounts of acetic acid (Table 6). No measurements were taken beyond day 14 because the Ermitage and Resi wines were blended at this stage. The Resi fermentations become more rapidly in 2011 than in 2010, beginning on the same day (or shortly after) the Qvevris were filled. However the fermentation process reached dryness in both years. The Ermitage must took longer to begin fermentation than Resi, starting 2 and 10 days later in 2010 and 2011, respectively.

## 4. Discussion

### 4.1. Isolation and Identification of Predominant Yeast Species

The isolation media we used enabled us to select different yeasts that were present in the winery environment and in wine musts undergoing spontaneous fermentation in steel tanks, thus favoring the detection and proliferation of some yeast species over others. Rose Bengal Chloramphenicol Agar (RBCA) medium was chosen instead of Sabouraud medium because the latter favored mold growth over yeasts (data not shown). Freezing the samples prior to analysis may have reduced the viability of the yeast although it is thought that this is a minor effect [26, 27]. Therefore, we acknowledge that yeast species present in low numbers are unlikely to be detected using this method, whereas abundant species are more likely to be recognized. Thus, only seven yeast species were isolated from the grape surface (*A. pullulans*, *C. magnus*, *F. floriforme*, *R. mucilaginosa*, *W. saturnus,* and *Z. florentinus*), with *A. pullulans* and *R. mucilaginosa* previously reported as colonizers of the grape surface [28]. A further 11 yeast species were isolated from vineyard air samples, all of which had previously been detected in winery environmental samples [28, 29]. The anamorphic yeast *Kloeckera apiculata*, previously reported as the predominant yeast species on the grape surface and in air samples [28], was not found in our investigation but instead the teleomorphic species *H. uvarum* was found in our environmental samples. 

We found that differences in yeast diversity were often dependent on the grape variety. This phenomenon can be attributed to several factors, including the different stages of berry ripening at harvest, physical damage to the grape surface, and pest management practices [29]. Although we studied different grape varieties grown in the same area and processed at the same winery, microclimatic conditions and viticultural practices may have influenced the yeast diversity we detected. 

Most of the yeasts isolated from the vineyard air were also present in the grape juice at the beginning of fermentation. All the yeasts identified in the cellar were also found later in the fermenting must. *R. mucilaginosa* was found in air samples from both the vineyard and the cellar, and on the grape surface, but not on the tank surface. During 2008, *Z. florentinus* was the only species found in all environmental samples (air and contact samples, from both the vineyard and the cellar). 

The viable counts of the environmental samples showed the presence of only non-*Saccharomyces* species. Although *S. cerevisiae* and related species such as *S. bayanus* are predominantly responsible for fermentation, they represent only a small fraction of the diversity we identified, which is consistent with other reports showing that *S. cerevisiae* is rarely isolated from natural sources such as berry and leaf surfaces when using viable count methods [30–33]. The small number of species isolated from the cellar environment (air and tank surface) during 2009 compared to 2008 may have been caused by the sanitary conditions adopted by the winery after the sampling results in 2008. The dynamic behavior of the yeast populations through the different stages of fermentation in steel tanks also differed among grape varieties. The detection of some yeast species only during the later stages of fermentation probably reflects their proliferation to cell numbers above the detection threshold of our assay rather than their genuine absence at the beginning of fermentation. The relative greater diversity of yeast species in red compared to white wines is consistent with the higher pH of red wines, providing favorable conditions for yeast growth [34]. In white wines, yeasts isolated from the grape skin were not found in the must, probably because they remained in the skin fraction during clarification, and this may also have contributed to the lower species diversity we observed.

The higher yeast diversity during the early stages of fermentation predominantly reflects the low ethanol tolerance of non-*Saccharomyces* species [3, 9, 10, 17, 35, 36]. Nevertheless, we found that non-*Saccharomyces* yeasts such as *P. klyveri*, *P. membranifaciens*, *R. mucilaginosa,* and *M. pulcherima* were active in the late fermentation stages in some must varieties. This is consistent with previous reports of ethanol tolerance in *M. pulcherima* [10, 35, 37], but *R. mucilaginosa* is usually found during the early stages of fermentation, and its presence along with the *Pichia* species later in fermentation could add complexity but also reduce the wine quality [34, 38]. 

Considering the results from the 2008 and 2009 harvests together, we observed that the generally higher yeast diversity in the must at the beginning of the fermentation was coincident with the rapid onset of the exponential phase. We evaluated the interrelation between the yeast species and the success of fermentation. We found that despite the diversity of yeasts in red and white varieties, white musts generally contained higher residual sugar levels than red musts and that sluggish fermentation was more likely. Such fermentations were characterized by the initial predominance of *C. zemplinina* and *S. bayanus*, as well as lower levels of *M. pulcherima* and *S. cerevisiae,* contrasting with the red wine musts. The impact of these properties on fermentation reflects the better performance of *S. cerevisiae* compared with the lower fructose uptake capacity of *S. bayanus* [39], which is consistent with our results. 

### 4.2. Dynamic Behavior of Wild Yeasts during Spontaneous Fermentation in Qvevris

We developed a novel qPCR method for the rapid, sensitive, and culture-independent detection of yeast species throughout fermentation, revealing that the non-*Saccharomyces* yeast *R. mucilaginosa* and *P. anomala* dominated the final stages of spontaneous fermentation in Qvevris. These results are important because non-*Saccharomyces *yeasts can influence the flavor and quality of wine in both positive and negative ways [40–42] despite their metabolic activity and abundance [19, 20, 43]. 

The diversity of the yeast species was variety dependent and vintage dependent, with *C. zemplinina* and *P. angusta* present only in the variety of Resi, and *P. kluyveri* present in both wines but only during the 2010 harvest. *H. uvarum* has previously been identified as the predominant species during the early stages of fermentation [9–11, 35] but we found no evidence for this species on the grape surface (viable cell count method) and found it was less prevalent during amphora fermentations (qPCR method). In contrast, *R. mucilaginosa* was found to be abundant in both the amphora and steel-tank fermentations using qPCR and culture-dependent methods, respectively. 

The Resi fermentations commenced almost immediately in 2011, even though similar numbers of yeast cells were present at the beginning of fermentation in both years, and *S. cerevisiae *was less abundant in 2011 than 2010. The minimal lag phase and rapid fermentation (completed in 3 days) could be explained by the climatic conditions in the weeks prior to harvest, which increased the temperature of the berries and the must after crushing (data not shown), favoring the rapid proliferation of *S. cerevisiae*. This suggests that berry temperature before pressing could play a key role in the success of spontaneous fermentation. We tested this hypothesis by studying parallel fermentations. Ermitage fermentations underwent a longer lag phase in 2011 (11 days) than 2010 (5 days, reaching dryness by day 14). During 2011, *R. mucilaginosa* and *P. anomala* were the predominant species throughout fermentation, and these are considered spoilage yeasts [44]. Several previous studies have shown that longer lag phases provide an opportunity for non-*Saccharomyces* yeasts and other microorganisms to outcompete beneficial microbes and produce toxic and/or noxious compounds, causing spoilage [45–49]. Accordingly, we found that 0.65 g L^−1^ acetic acid was produced in this fermentation, which is above the upper range in normal wines and is considered undesirable [8, 50, 51]. 

Despite the presence of spoilage yeast, the success of spontaneous fermentation seems to correlate with the length of the lag phase, since fermentations with a longer lag phase were more likely to fail. The onset of fermentation also depended on the temperature of the must, so this is a key factor to consider when predicting the outcome of a spontaneous fermentation. 

Our integration of novel analytical methods with traditional winemaking using Qvevris provides the basis for further experiments to determine the influence of Qvevris on spontaneous fermentation. Comparative studies with steel-tank fermentations, using the same raw materials (grape variety and harvest year), should be carried out to investigate the impact of Qvevris in more detail.

## 5. Conclusions

The predominant yeasts found in the winery (i.e., *Metschnikowia pulcherima*, *Rhodotorula mucilaginosa,* and some *Pichia* species) were used as a basis for the development of an antibody chip for the identification and semiquantitative detection of wild yeast. The effect of the initial yeast concentration and the berry/must temperature on the length of the fermentation lag phase and thus the quality of spontaneous fermentation will be investigated in more detail to improve the performance of this device. We have also provided the first quantitative evidence describing the dynamic behavior of yeast populations during spontaneous fermentation in amphora vessels. 

## Figures and Tables

**Figure 1:** Yeast population recovered at the end of spontaneous fermentation in steel tanks during the 2008 and 2009 harvest seasons.

**Figure 2:** Spontaneous fermentation profile, expressed in g L^−1^, for the white grape varieties in stainless steel tanks during the 2008 and 2009 harvest seasons. (a) Pinot Noir; (b) Cornalin; (c) Chardonnay; (d) Petit Arvine; (e) Gutedel.

**Figure 3:** Dynamic behavior of wild yeast populations during the spontaneous fermentation of Ermitage grapes in Qvevris, measured by qPCR: (a) 2010 harvest; (b) 2011 harvest.

**Figure 4:** Dynamic behavior of wild yeast populations during the spontaneous fermentation of Resi grapes in Qvevris, measured by qPCR: (a) 2010 harvest; (b) 2011 harvest.

**Figure 5:** Spontaneous fermentation profile in Qvevris during the 2010 and 2011 harvests: (a) Ermitage; (b) Resi.

**Table 1:** Grape varieties used for the analysis of dynamic wild yeast populations during spontaneous fermentation in stainless steel tanks and Qvevris.

	Harvest		
	2008-2009 (steel tank)		2010-2011 (Qvevris)
	Pinot Noir (R)	Chardonnay (W)	Resi (W)
Grape variety	Cornalin (R)	Petit Arvine (W)	Ermitage (W)
		Gutedel (W)	

(R): red variety; (W): white variety.

**Table 2:** Specific primers used for qPCR analysis.

Yeast species	Primer name	Primer sequence	Product size	Annealing temperature °C
*Candida zeylanoides *	CZ-5fw	5′-CGATGAGATGCCCAATTCCA-3′	191 bp	58
	CZ-3bw	5′-GAAGGGAACGCAAAATACCAA-3′		
*Zygosaccharomyces florentinus *	ZF-5fw	5′-CTTGAGCTCCTTGTAAAGC-3′	256 bp	55
	ZF-3bw	5′-CTAGGTTTTCTGCTGCCG-3′		
*Metschnikowia pulcherrima *	MP-5fw	5′-CAACGCCCTCATCCCAGA-3′	253 bp	60
	MP-3bw	5′-AGTGTCTGCTTGCAAGCC-3′		
*Williopsis saturnus *	WS-5fw	5′-GGGTGTCCAGTGCTTTG-3′	199 bp	56
	WS-3bw	5′-CCCAAGAAGGGAAGATAATCAC-3′		
*Pichia kluyveri *	PK-5fw	5′-AGTCTCGGGTTAGACGT-3′	169 bp	55
	PK-3bw	5′-GCTTTTCATCTTTCCTTCACA-3′		
*Rhodotorula mucilaginosa *	RM-5fw	5′-GCGCTTTGTGATACATTTTC-3′	169 bp	54
	RM-3bw	5′-CCATTATCCATCCCGGAAAA-3′		
*Pichia angusta *	PANG-5fw	5′-GTGTCCATTTCCGTGTAAGA-3′	175 bp	56
	PANG-3bw	5′-AGCCCACCCACAAG-3′		
*Pichia anomala *	PA-5fw	5′-ACGTCATAGAGGGTGAGAAT-3′	197 bp	57
	PA-3bw	5′-AAACACCAAGTCTGATCTAATG-3′		
*Candida glabrata *	CG-5fw	5′-GAGGGTGTCAGTTCTTTGT-3′	224 bp	56
	GC-3bw	5′-GTGAGCTGCGAGAGTC-3′		
*Hanseniaspora uvarum *	HU-5fw	5′-GGCGAGGGATACCTTTTCTCTG-3′	172 bp	59
	HU-3bw	5′-GAGGCGAGTGCATGCAA-3′		
*Pichia fermentans *	PF-5fw	5′-TTGCCTATGCTCTGAGGCC-3′	170 bp	61
	PF-3bw	5′-TCCATGTCGGGCGCAAT-3′		
*Saccharomyces cerevisiae *	SC-5fw	5′-AGGAGTGCGGTTCTTTCTAAAG-3′	215 bp	59
	SC-3bw	5′-TGAAATGCGAGATTCCCCCA-3′		
*Torulaspora delbrueckii *	TD-5fw	5′-GTGGCGAGGATCCCAG-3′	186 bp	58
	TD-3bw	5′-CTATCGGTCTCTCGCAA-3′		

**Table 3:** Sizes of digested and undigested nested PCR products representing different yeast species derived using the T-RFLP method.

Yeast species	Size (bp)	
	Nested PCR	Digested
Aureobasidium pullulans*	254	—
Botryotinia fuckeliana*	—	223
*Bulleromyces albus *	195	164
*Candida glabrata *	478	224
*Candida zemplinina *	200	
*Candida zeylanoides *	269	238
*Cryptococcus flavus *	169	134
*Cryptococcus magnus *	211	—
*Dekkera bruxellensis *	168	134
Epicoccum nigrum*	216	—
*Filobasidium floriforme *	237	204
*Hanseniaspora guilliermondii *	364	66
*Hanseniaspora uvarum *	365	66
*Hyphopichia burtonii *	159	124
*Issatchenkia orientalis *	178	148
*Kluyveromyces lactis *	305	273
*Metschnikowia pulcherrima *	140	107
*Metschnikowia sp. *	348	—
*Pichia angusta *	379	351
*Pichia anomala *	258	228
*Pichia fermentans *	156	122
*Pichia holstii *	—	248
*Pichia kluyveri *	162	128
*Pichia membranifaciens *	165	130
*Rhodotorula mucilaginosa *	229	198
*Saccharomyces bayanus *	435	405
*Saccharomyces cerevisiae *	441	410
*Saccharomyces pastorianus *	435	405
*Sporidiobolus pararoseus *	222	197
*Torulaspora delbrueckii (wild yeast isolate) *	370	340
*Williopsis saturnus *	252	134
*Zygosaccharomyces florentinus *	244	213

*Molds.

**Table 4:** Yeasts isolated from the winery environment during the 2008 and 2009 harvest seasons.

Yeast species	Air vineyard		Air cellar		Tank surface		Grape surface*	
	2008	2009	2008	2009	2008	2009	2008	2009
*Aureobasidium pullulans *		+					Gu	Gu
*Bulleromyces albus *	+	+						
*Candida zemplinina *		+						
*Cryptococcus magnus *		+						Gu
*Filobasidium floriforme *							Ch	Ch, Pa, Gu
*Hanseniaspora uvarum *		+			+			
*Metschnikowia pulcherrima *	+		+					
*Pichia angusta *								
*Pichia anomala *	+				+			Co
*Pichia kluyveri *	+		+					
*Rhodotorula mucilaginosa *	+		+			+	Pn	Pa, Gu
*Sporidiobolus pararoseus *	+	+						
*Williopsis saturnus *								Pa
*Zygosaccharomyces florentinus *	+		+		+		Ch	Co

*Varieties of grapes and musts: Pinot Noir (Pn); Cornalin (Co); Chardonnay (Ch); Petite Arvine (Pa); Gutedel (Gu).

**Table 5:** Yeasts found during spontaneous fermentation in stainless steel tanks, during the 2008 and 2009 harvest seasons.

Yeast species	Grape variety				
	Pinot Noir	Cornalin	Chardonnay	Petit Arvine	Gutedel
*Bulleromyces albus *					a
*Candida zemplinina *		a	a; b	a	a
*Candida zeylanoides *					a
*Candida Krusei or Issatchenkia orientalis *		a	a		
*Cryptococcus flavus or Dekkera bruxellensis *					a
*Filobasidium floriforme *					a
*Hanseniaspora uvarum *	a; b	a	a		
*Metschnikowia pulcherrima *	a; b; c	a; b; c	a; b; c	a	a
*Pichia anomala *	a	a	a		
*Pichia burtonii *		a			
*Pichia holstii *		a			
*Pichia kluyveri *	a	a; c	a		a
*Pichia membranifaciens *			a; b; c	a	
*Rhodotorula mucilaginosa *	c		a	a	a
*Saccharomyces bayanus *	a; b; c	a, b; c	a; b; c	a, b; c	a, b; c
*Saccharomyces cerevisiae *	a; b; c	a	a; b; c	a; c	a
*Sporidiobolus pararoseus *	b	a			
*Torulaspora delbrueckii *	a	a	a	a	a
*Zygosaccharomyces florentinus *			a		a

a: detected at the beginning of the fermentation; b: detected during log phase; c: detected during stationary phase.

**Table 6:** Acetic acid production in the spontaneous fermentations.

Fermentation vessel	Variety	Harvest season	Acetic acid (mg L^−1^)
	Pinot Noir	2008	65.61 ± 2.5
		2009	154.69 ± 23.48
	Cornalin	2008	150.71 ± 18.62
		2009	145.0 ± 7.07
Steel tanks	Chardonnay	2008	154.64 ± 91.43
		2009	379.15 ± 0
	Petite Arvine	2008	131.64 ± 76.88
		2009	280.0 ± 0
	Gutedel	2008	24.93 ± 0
		2009	94.0 ± 39.0

Qvevri	Resi	2010	180.0 ± 0
		2011	270.0 ± 10.0
	Ermitage	2010	160.0 ± 30.0
		2011	650 ± 20.0

**Table 7:** Yeasts identified by qPCR during spontaneous fermentations in Qvevris during the 2010 and 2011 harvest seasons.

Yeast species	Resi		Ermitage	
	2010	2011	2010	2011
*Candida zemplinina *	a; b; c	b		
*Metschnikowia pulcherima *	a; b; c	a; b; c	a; b; c	a; b; c
*Williopsis saturnus *	a; c	a		b; c
*Pichia kluyveri *	a		b	
*Rhodotorula mucilaginosa *	a; b; c	a; b; c	a; b; c	a; b; c
*Pichia angusta *	b	c		
*Pichia anomala *	a; b; c	a; b; c	a; b; c	a; b; c
*Hanseniaspora uvarum *	a; b; c	a; b; c	a; b; c	a; b; c
*Saccharomyces cerevisiae *	a; b; c	a; b; c	a; b; c	a; b; c
*Torulaspora delbrueckii *	a; b; c	a; b; c	a; b; c	a; b; c

a: detected at the beginning of the fermentation; b: detected during log phase; c: detected during stationary phase.
